# Bayesian Analysis of Trends in Utilization of Maternal Healthcare Services in Pakistan during 2006-2018

This article has been retracted.

**DOI:** 10.1155/2021/4691477

**Published:** 2021-11-27

**Authors:** Navid Feroze, Muhammad Ajmal Ziad, Rabia Fayyaz, Yaé Ulrich Gaba

**Affiliations:** ^1^Department of Statistics, The University of Azad Jammu and Kashmir, Muzaffarabad, Pakistan; ^2^COMSATS University Islamabad, Islamabad, Pakistan; ^3^Quantum Leap Africa (QLA), AIMS Rwanda Centre, Remera Sector KN 3, Kigali, Rwanda

## Abstract

**Objectives:**

This study is aimed at investigating the time trends and disparities in access to maternal healthcare in Pakistan using Bayesian models. *Study Design*. A longitudinal study from 2006 to 2018.

**Methods:**

The detailed analysis is based on the data from Pakistan Demographic and Health Survey (PDHS) conducted during 2006-2018. We have proposed Bayesian logistic regression models (BLRM) to investigate the trends of maternal healthcare in the country. Based on different goodness-of-fit criteria, the performance of proposed models has also been compared with repeatedly used classical logistic regression models (CLRM).

**Results:**

The results from the analysis suggested that BLRM perform better than CLRM. The access to antenatal healthcare increased from 61% to 86% during years 2006-18. The utilization of medication also improved from 44% in 2006 to 60% in 2018. Despite the improvements from 2006 to 2018, every three out of ten women were not protected against neonatal tetanus, neither delivered in the health facility place nor availed with the skilled health provider at the time of delivery during 2018. Similarly, two-fifth mothers did not received any skilled postnatal checkup within two days after delivery. Additionally, the likelihood of MHS provided to mothers is in favor of mothers with lower ages, lower birth orders, urban residences, higher education, higher wealth quintiles, and residents of Sindh and Punjab.

**Conclusions:**

The gaps in utilization of MHS in different socioeconomic groups of the society have not decreased significantly during 2006-2018. Any future maternal health initiative in the country should focus to reduce the observed disparities among different socioeconomic sectors of the society.

## 1. Introduction

According to the report of the World Health Organization (WHO), approximately 800 maternal deaths are witnessed daily [1]. Hence, maternal mortalities remained the global healthcare challenge. Reducing the proportion of maternal mortalities is one of the important goals of Sustainable Development Goals (SDG) 2015. Being signatory of the SDGs 2015-30, Pakistan has taken some initiatives, such as installation of National Maternal, Neonatal and Child Health program, to foster the delivery of maternal healthcare in the country. However, there is still lack of accessibility to MHS in Pakistan, and various socioeconomic factors are responsible for this deprivation [2]. There have been many studies in Pakistan exploring the important determinants of MHS in the country. The utilization of antenatal care (ANC) and postnatal care (PNC) has been found to be the most important in reducing the maternal mortalities [3, 4]. However, utilization of these services in Pakistan is quite low [5]. There have been many factors hindering the delivery of these services in the country such as poverty [2, 6], lower education [7, 8], high transport costs and conventional attendants [9, 10], higher birth orders [2], rigidly structured caste hierarchy [11], attitude of communities and health system in rural areas [12], and low knowledge about maternal health among fertile women [7]. However, only few of these studies considered the nationally represented datasets. The continuous analysis of trends for utilization of maternal healthcare services, using nationally representative data, is necessary to plan and implement the strategies accordingly for better delivery of these services.

There are few interesting studies regarding the investigation of trends in delivery of maternal healthcare in developing counties such as for India [13], China [14], Ethiopia [15], and Cambodia [16]. However, there is a dearth of such studies in Pakistan. A careful review of the literature suggests only two recent studies investigating the trends related to MHS in Pakistan. One of these studies has investigated the tendencies of caesarean section deliveries in the country with respect to time [17]. Another contribution has compared the data from two PDHS conducted in 2012-13 and 2017-18 to explore the role spousal violence in poor maternal healthcare utilization in the country [18]. There is still a need of detailed studies analyzing the differentials in the delivery of MHS across various demographic and socioeconomic sectors of the society.

In addition, almost all the recent contributions regarding analysis of MHS in Pakistan have utilized classical models for investigation of the important determinants of maternal healthcare in the country. On the other hand, some of the studies have explored that the Bayesian methods often produce better results as compared to classical methods [19–21]. The main feature of Bayes methods is that they allow us to incorporate the prior information regarding the parameters of the concerned models. The inclusion of prior information updates the current information about the model parameters [22]. The Bayesian methods are applicable when the parametric estimates correlated [23, 24], which is not the case for many classical methods. It is worth mentioning here that classical methods mostly rely on the maximum likelihood estimation (MLE). However, in small samples, the asymptotic properties for MLE are often not fulfilled, which creates serious inferential issues for MLE [25]. Further, the interval estimation is very important in health sciences research, and Bayesian estimation provides very commonsense interpretation for the interval estimation [22]. These merits of the Bayesian methods have attracted many researchers to use these methods in different fields of applications [26]. The said methods have provided the improved estimation (as compared to classical methods) of individual risk of type II diabetes using multiple informant family health history [27]. The Bayesian methods have also been proved to be better than classical methods in analyzing the utilization of ANC in Ethiopia [28]. The said Bayesian methods have also provided efficient results for analyzing the important determinants of maternal health care in Ghana [29], India [30], Nigeria [31], and Ethiopia [25, 32]. However, to the best of our knowledge, the Bayes methods have not yet been used to analyze the utilization of MHS in the country.

We have conducted this study to explore the changes (over time) occurring in utilization of MHS across different demographic and socioeconomic sectors of the society. Due to added advantages of BLRM, these models have been proposed for the statistical analysis in the study. The performance of the CLRM and BLRM has been compared using two goodness-of-fit criteria, namely, Akaike information criteria (AIC) and Bayesian information criteria (BIC). The data from three PDHS were used for analysis. These surveys were conducted during 2006-07, 2012-13, and 2017-18, respectively. The results from the study explored the improved performance of MLRM as compared to CLRM. The study also identified the disparities in delivery of MHS in the country across various socioeconomic groups. Unfortunately, the observed inequalities among different socioeconomic sections of society continued to persist during the study period.

## 2. Methods

The data have been obtained from the published reports of PDHS conducted in years 2006-07, 2012-13, and 2017-18, respectively. The information has been obtained from the mothers lying in the age group 15-49 years. Two-stage stratified sample design has been used to collect the information in each PDHS. In the first stage, the enumeration blocks were selected with probability proportional to size. In the second stage, the systematic sampling was used to select the required number of households for the inquiry. The pretesting was used to improve the survey method. The main surveys were carried out using sample size 10,023 for PDHS 2006-07, 13,558 for PDHS 2012-13, and 14,161 for PDHS 2017-18. However, the information on coverage of ANC, use of medical drugs during pregnancy, and protection against neonatal tetanus was asked from the mothers aged 15-49 years for their pregnancy for the most recent live birth in five years prior to this survey. This information was collected from 5678, 7446, and 6710 eligible women for the PDHS surveys conducted in 2006-07, 2012-13, and 2017-18, respectively. On the other hand, the responses on delivery in health facility and delivery by skilled provider contained the information regarding all live births in the last five years before the corresponding survey. For these factors, 9122, 11977, and 10494 eligible women were interviewed in 2006-07, 2012-13, and 2017-18, respectively. Finally, information regarding postnatal checkup was asked from women having live births in two years before the respective survey. In this case, 5678, 4245, and 3936 eligible women were interviewed in 2006-07, 2012-13, and 2017-18, respectively. The response rates for PDHS conducted in 2006-07, 2012-13, and 2017-18 were 95%, 93%, and 94%, respectively. The survey methodologies were approved by the National Institute of Population Studies, Islamabad, Pakistan. Since the data from published reports of PDHS have been used for analysis, the ethical approval from the concerned institutes was not required.

A careful review of literature suggests that all of the earlier contributions considered the classical methods, such as logistic regression, for the analysis of MHS in Pakistan. Further, the literature contains very few studies based on nationally representative data. The earlier contributions using nationally representative data have considered quite lower number of response variables to reach the conclusions. We have proposed the BLRM to identify the important determinants of MHS in Pakistan. The proposed models have been compared with most repeatedly used classical models, such as CLRM. These comparisons have been carried out using values of different goodness-of-fit criteria, namely, AIC and BIC. The detailed analysis contain different response variables such as (i) antenatal care coverage (ANC), (ii) use of medical drugs during pregnancy (MDDP), (iii) protection against neonatal tetanus (PANT), (iv) delivery in health facility place (DAHFP), (v) delivery by a skilled provider (DBSP), (vi) postnatal checkup during the first two days of delivery (PCWTD), and (vii) skilled postnatal checkup during the first two days of delivery (SPCWTD). On the other hand, mother's age at birth (MAB), birth order (BO), residence (RES), mother's education level (ME), wealth quintile (WQ), and region (REG) of the respondents have been considered as exploratory variables in the study. We have merged the original classification of the explanatory variables for the cause of brevity. We have specified our study to compare the two extreme ends of the classifications. Moreover, the change in receipt of maternal healthcare, in Pakistan from 2006 to 2018, has been analyzed using CLRM and BLRM. The stepwise forward selection method was used for the variable selection. Only the significant explanatory variables were included in the proposed model. All the results have been obtained using R software.

## 3. Bayesian Regression Model

Assuming the likelihood contribution of the *i*^th^ subject in the logistic regression model as binomial, the likelihood function for the subjects can be written as

(1) $$\begin{array}{c} {\text{likelihood}}_{i}=\pi {\left(x_{i}\right)}^{y_{i}}{\left\{1-\pi \left(x_{i}\right)\right\}}^{1-y_{i}}, \end{array}$$

where *π*(*x*_*i*_) represents the probability of the event for the subject *i* who has covariate vector *x*_*i*_ and *y*_*i*_ indicates the presence, *y*_*i*_ = 1, or absence *y*_*i*_ = 0 of the event of that subject.

(2) $$\begin{array}{c} \pi \left(x\right)=\frac{e^{\beta_{0}+\beta_{1}X_{1}+\cdots +\beta_{p}X_{p}}}{1+e^{\beta_{0}+\beta_{1}X_{1}+\cdots +\beta_{p}X_{p}}}. \end{array}$$

Now, the normal prior has been assumed for the parameters of model (2), which is of the form

(3) $$\begin{array}{c} \beta_{j}\sim N\;\left(\mu_{j},{\sigma_{j}}^{2}\right),\;\;j=0,1,2,\cdots ,p. \end{array}$$

The posterior distribution is derived by multiplying the prior distribution over all parameters by the full likelihood function

(4) $$\begin{array}{c} \text{Posterior}=\overset{n}{\underset{i=1}{\prod }}\left[{\left(\frac{e^{\beta_{0}+\beta_{1}X_{\text{i}1}+\cdots +\beta_{p}X_{ip}}}{1+e^{\beta_{0}+\beta_{1}X_{i1}+\cdots +\beta_{p}X_{ip}}}\right)}^{y_{i}}{\left(1-\frac{e^{\beta_{0}+\beta_{1}X_{i1}+\cdots +\beta_{p}X_{ip}}}{1+e^{\beta_{0}+\beta_{1}X_{i1}+\cdots +\beta_{p}X_{ip}}}\right)}^{\left(1-y_{i}\right)}\right]\times \;\overset{p}{\underset{j=0}{\prod }}\frac{1}{\sqrt{2\pi \sigma_{j}}}\exp\left\{\frac{1}{2}{\left(\frac{\beta_{j-}\mu_{j}}{\sigma_{j}}\right)}^{2}\right\}. \end{array}$$

## 4. Results

This section includes the numerical results regarding analysis of MHS in the country. The descriptive results have been reported in Table 1. The comparison between BLRM and CLRM using amounts of AICs and BICs has been presented in Table 2. The ORs for different response variables using BLRM have been reported in Tables 3 and 4. The results given in Table 1 suggest that the access to ANC increased from 61% to 86% during years 2006-18 in the country. The utilization of medication also improved from 44% in 2006 to 60% in 2018. Despite the improvements from 2006 to 2018, every three out of ten women were not protected against neonatal tetanus, neither delivered in the health facility place nor availed the skilled health provider at the time of delivery during 2018. Similarly, two-fifth mothers did not received any skilled postnatal checkup within two days after delivery.

The detailed comparison of classical and BLRM based on values of AIC and BIC have been reported in Table 2. The lower values of AIC and BIC for BLRM suggest the better performance of BLRM as compared to CLRM. Hence, we have reported the detailed results under BLRM only.

Table 3 reports the analysis of different response variables using two categories of predictors under BLRM. This analysis has been carried out in order to observe the gap/inequalities in utilization of the MHS in country falling in the lowest and highest order of their classification. For example, MAB was an original category in three groups less than twenty years, twenty to thirty-four years, and thirty-five to forty-nine years. However, we have considered only two groups below thirty-five years and thirty-five and above years. Similarly, BO was categorized in two groups: (i) first birth and (ii) second and higher births. The ME was divided into two classes, namely, (i) no education and (ii) primary to higher education. Finally, the WQ was classified as (i) lowest wealth quintile and (ii) second to highest wealth quintile. The classifications were made for the cause of brevity.

Table 3 reveals that the ORs for ANC are inclined to mothers with lower ages. For example, the OR for mother's age group 35-49 years, as compared to the age group below 35 years, was 0.556 {0.496, 0.626}^d^ in 2006-07 which decreased to 0.497 {0.442, 0.557}^d^ in 2012-13 and further decreased to 0.495 {0.427, 0.576}^d^ in 2017-18. The availability of ANC drastically increased over time in favor of mothers with lower birth orders. For example, the corresponding OR for first birth order as compared to higher birth orders increased from 1.966 {1.726, 2.239}^d^ in 2006-07 to 2.743 {2.265, 3.332}^d^ in 2017-18. As far as the comparison of ANC for the mothers belonging to urban and rural areas are concerned, a steady increase in the availability of the said services in urban areas is observed. This can be seen from the fact that the corresponding OR in favor of urban mothers was 3.097 {2.786, 3.471}^d^ in 2006-07 which increased to 3.609 {3.090, 4.269}^d^ in 2017-18. Similarly, the ORs in favor of mothers with high education levels increased exponentially from 17.385 {11.370, 29.400}^d^ in 2006-07 to 32.406 {17.359, 76.161}^d^ in 2017-18. Further, the said ORs also increased significantly in favor of mothers with high incomes. The corresponding OR in 2006-07 was 9.635 {7.979, 11.778}^d^ which increased to 10.871 {7.716, 15.865}^d^ in 2017-18. Similar trends can be seen from Figure 1(a). The results from the analysis under classical logistic regression models have been reported in Table 5. The results in ANC using complete categories of the explanatory variables have been reported in Table 6. Letters b, c, and d attached the 95% confidence intervals for the ORs suggest the statistical significance of the corresponding ORs. From the results, we can see almost all the ORs are significant at 5% level of significance.

The results from Table 3 also suggest that younger mothers are more likely to use the MDDP, and this trajectory seems to persist over time. This can be seen from the fact that corresponding OR in favor of women falling in the age group 35-49 years, as compared to those aged below 35 years, was 0.608 {0.538, 0.689}^d^ in 2006-07 which slightly increased to 0.687 {0.607, 0.817}^b^ in 2017-18. Similarly, the likelihood of using the MDDP remained in favor of mothers with first birth order during 2006-18 in the country. For example, the OR for first birth order, as compared to higher birth orders, increased from 1.445 {1.289, 1.621}^d^ in 2006-07 to 1.515 {1.363, 1.680}^d^ in 2017-18. However, the usage of MDDP seems to have improved for the mothers from rural areas, having no education and falling in lowest wealth quintiles. This is due to the fact that the corresponding ORs in favor of mothers from urban areas, having primary to higher education and falling in the higher wealth quintiles have decreased over time.  Figure 1(b) also suggests the similar patterns. Table 3 and Figure 1(c) also suggest that tendency of PANT is relatively higher for mothers with lower ages, lower birth orders, urban residents, higher education, and higher wealth quintile. Similarly, from Table 3 and Figures 1(d)–1(g), it can be assessed that mother's age, birth order, residence, education, and wealth were significantly related to DAHFP, DBSP, PCWTD, and SPCWTD in case of each PDHS.

The results reported in Table 4 suggest that the delivery of ANC, MDDP, DAHFP, DBSP, PCWTD, and SPCWTD is higher in Sindh as compared to other provinces of the country. On the other hand, the mothers from Punjab are more likely to have PANT. The delivery of MHS is least in Balochistan and KPK.

## 5. Discussion

The results from the study suggest that the BLRM can be used as an improved alternative to the CLRM in analyzing the maternal health services. The study also explored that mother's age, birth order, residence, education, wealth, and region contribute significantly in delivery of MHS in Pakistan [33, 34]. Mother's education and wealth were identified to be the most dominant factors in access to MHS in the country [2, 17]. The delivery of MHS was higher for younger mothers [35–37]. The behavior of inequalities in utilization of MHS among younger and elder mothers was uniform over the study period. Similarly, the access to MHS was significantly higher at first birth as compared to higher births. The gap in utilizing the MHS with respect to birth order has even increased (over time) for majority of response variables. This simply indicates that mothers provided with more care at the time of first birth. This may be interpreted as psychological factor because the parameters and family are often more excited about the first baby, and unfortunately, the subsequent babies often not received the desired attention [2]. The residence of the mothers was observed to be the third most dominant factor in delivery of MHS in the country. The access to MHS was at least two times more for urban areas as compared to rural areas in the country. Unfortunately, the disparity in delivery of MHS with respect to residence continued from 2006 to 2018 in the country. Similarly, the inequalities in provision of MHS among different provinces of the country also persisted during 2006 to 2018. The use of MHS was drastically low in KPK and Balochistan as compared to Punjab. The financial status of the families was found as the second most prominent contributor in delivery of MHS in the country. The mothers belonging to families falling in lowest wealth quintiles are receiving severely low MHS as compared to those falling in higher wealth quintiles [38, 39]. The inequalities in usage of MHS with respect to financial status remained almost constant during the study period. Similarly, the delivery of MHS was least for illiterate mothers [2, 40–44]. The gap in utilization of MHS was the most with respect to education of the mothers. The said gap has even increased (over time) for some factors, namely, ANC and PCWTD. However, it was encouraging to observe that access to MDDP, PANT, DAHFP, DBSP, and SPCWTD improved for illiterate mothers during the study period.

In summary, it can be shown that the ORs for different factors regarding MHS in Pakistan have increasing trend for the mothers with lower birth orders. On the other hand, the ORs for the most of the factors have not change a lot with respect to residence and wealth of the concerned families. Also, the gap between the availability of MHS to urban and rural residents, educated and noneducated mothers, and mothers from higher and lower wealth quintiles is significant and steady. All possible resource should be mobilized to minimize these disparities. An additional issue is that the ORs, for the majority of the said factors, have been decreasing in all the provinces of the country, as compared to Punjab. Especially the situation in KPK and Balochistan is quite miserable. Hence, all the stakeholders should start an aggressive campaign to bridge up this elevating gap.

The results from the study are in close agreement with earlier studies conducted in Pakistan. For example, some contributions [2, 33, 34] indicate that mothers' age, birth order, residence, education level, wealth, and region are highly associated with availability of MHS in the country. Additionally, the findings of the study are also in accordance with earlier studies conducted in other developing countries. For example, the previous studies conducted in developing countries such as Nepal [38], Bangladesh [39], Nigeria [40], India [41–43], and Ethiopia [44] also concluded that mothers with higher levels of education and wealth are more likely to use maternal and child health services. Similarly, the studies conducted in Turkey [35], Mali [36], and Zimbabwe [37] have explored that elder women are less likely to utilize the maternal healthcare.

## 6. Strengths and Limitations of the Study

The BLRM have been proposed for exploring the trends of inequalities in utilization of MHS across different socioeconomic sectors of society in Pakistan. The proposed models provided improved estimation as compared to repeatedly used CLRM. The study has used nationally representative data from different PDHS conducted during 2006 to 2018. The data has been collected using a comprehensive methodology under strict technical and ethical considerations which have increased the validity of the results. In addition, the study contains more detailed analysis than the earlier studies by incorporating seven response variables for analysis. Nonetheless, the study was not free from limitations. The main source of information was mother's self-reporting. Hence, the social desirability biases might have been included. Since the information was asked from the mothers regarding latest birth, the information on utilization of MHS during earlier births remained unknown. In order to counter the said limitations of the study, the future PDHS may ask the information from the mothers about their earlier births as well. The social desirability biases can be reduced by using neutrally worded questions, indirect questions, and use of both stated and derived questioning.

## 7. Conclusion

The maternal healthcare is Sustainable Development Goal (SDG) number three. Being signatory of the SDGs 2015-30, Pakistan has taken some initiatives, such as installation of National Maternal, Neonatal and Child Health program, to foster the delivery of maternal healthcare in the country. Keeping in view the importance of the issue, number of researchers has conducted the studies to investigate the important determinant of MHS in the country and to identify the inequalities in delivery of MHS among various socioeconomic sectors of the society. However, all the earlier studies considered the classical models for analysis in the country. In addition, there is still need to investigate the change in utilizations of the MHS in the country over time.

We have proposed BLRM to explore the trends of inequalities regarding utilization of MHS among different socioeconomic groups of the society. The performance of proposed models has been compared with frequently used CLRM using different goodness-of-fit criteria such as AIC and BIC. The performance of BLRM was observed to be better than CLRM. The results based on BLRM advocated that the likelihood of MHS was higher for the mothers with lower ages, lower birth order, urban residence, higher education level, higher wealth quintile, and residence of Sindh and Punjab. The access of MHS was highly dependent on education followed by wealth, residence, birth order, and age at birth. Though the initiatives taken by the government have resulted in overall improvement in the availability of the MHS in the country, the inequalities in delivery of MHS among different socioeconomic sectors of the society are still persisting. The policy maker should plan and implement the strategies to reduce the observed disparities in availability of the MHS for different sectors of society.

## Figures and Tables

**Figure 1:** Comparison of ORs for different output variables over time using Bayesian logistic regression model.

**Table 1:** Percentage distribution for availability of MHS for each outcome variables over the time.

Factors	Yes	No	Total
*2006-07*			
ANC	3459 (61%)	2219 (39%)	5678
Medical drugs during pregnancy	2478 (44%)	3200 (56%)	5678
Protection against neonatal tetanus	3396 (60%)	2282 (40%)	5678
Health facility place	3126 (34%)	5996 (66%)	9122
Skilled provider	3541 (39%)	5581 (61%)	9122
Checkup during 2 days	2239 (39%)	3439 (61%)	5678
Skilled postnatal checkup	1518 (27%)	4160 (73%)	5678
*2012-13*			
ANC	5441 (73%)	2005 (27%)	7446
Medical drugs during pregnancy	3516 (47%)	3930 (53%)	7446
Protection against neonatal tetanus	4758 (64%)	2688 (36%)	7446
Health facility place	5775 (48%)	6202 (52%)	11977
Skilled provider	6242 (52%)	5735 (48%)	11977
Checkup during 2 days	2559 (60%)	1686 (40%)	4245
Skilled postnatal checkup	2031 (48%)	2214 (52%)	4245
*2017-18*			
ANC	5783 (86%)	927 (14%)	6710
Medical drugs during pregnancy	4047 (60%)	2663 (40%)	6710
Protection against neonatal tetanus	4623 (69%)	2087 (31%)	6710
Health facility place	6942 (66%)	3552 (34%)	10494
Skilled provider	7277 (69%)	3217 (31%)	10494
Checkup during 2 days	2425 (62%)	1511 (38%)	3936
Skilled postnatal checkup	2238 (57%)	1698 (43%)	3936

**Table 2:** Amounts of AICs and BICs under classical logistic regression models for ANC.

Factors	Classical models				Bayesian models			
	2006-07		2017-18		2006-07		2017-18	
	AIC	BIC	AIC	BIC	AIC	BIC	AIC	BIC
ANC	17.708	15.095	17.210	14.676	15.737	13.384	15.668	12.933
MDDP	17.670	15.056	17.740	15.142	15.758	13.333	15.905	13.448
PANT	17.709	15.096	17.732	15.138	15.971	13.667	15.827	13.593
DAHFP	18.619	16.005	18.653	16.062	16.546	14.192	16.982	14.155
DBSP	18.702	16.088	18.623	16.041	16.041	13.934	16.309	13.862
PCWTD	17.617	15.003	16.824	14.274	16.171	13.549	15.039	12.959
SPCWTD	17.330	14.716	16.828	14.255	15.266	13.674	14.762	12.704

^∗^AIC: Akaike information criteria; BIC: Bayesian information criteria; ANC: antenatal care coverage; MDDP: use of medical drugs during pregnancy; PANT: protection against neonatal tetanus; DAHFP: delivery in health facility place; DBSP: delivery by a skilled provider; PCWTD: postnatal checkup during the first two days of delivery; SPCWTD: skilled postnatal checkup during the first two days of delivery.

**Table 3:** Comparison of ORs regarding different response variables for years 2006-18 using BLRM.

Response variables	Explanatory variables	PDHS 2006-07	PDHS 2012-13	PDHS 2017-18
		OR (95% CI for OR)	OR (95% CI for OR)	OR (95% CI for OR)
ANC	MAB	0.556 {0.496, 0.626}^d^	0.497 {0.442, 0.557}^d^	0.495 {0.427, 0.576}^d^
	BO	1.966 {1.726, 2.239}^d^	2.238 {1.970, 2.552}^d^	2.743 {2.265, 3.332}^d^
	RES	3.097 {2.786, 3.471}^d^	3.597 {3.205, 4.041}^d^	3.609 {3.090, 4.269}^d^
	ME	17.385 {11.370, 29.400}^d^	14.265 {10.026, 21.434}^d^	32.406 {17.359, 76.161}^d^
	WQ	9.635 {7.979, 11.778}^d^	13.265 {10.367, 17.258}^d^	10.871 {7.716, 15.865}^d^

MDDP	MAB	0.608 {0.538, 0.689}^d^	0.742 {0.664, 0.831}^d^	0.687 {0.607, 0.817}^b^
	BO	1.445 {1.289, 1.621}^d^	1.539 {1.397, 1.697}^d^	1.515 {1.363, 1.680}^d^
	RES	2.454 {2.223, 2.704}^d^	2.112 {1.935, 2.292}^d^	1.658 {1.519, 1.812}^d^
	ME	6.956 {5.497, 8.957}^d^	5.121 {4.324, 6052}^d^	3.935 {3.399, 4.595}^d^
	WQ	4.601 {4.061, 5.219}^d^	3.321 {2.975, 3.725}^d^	3.491 {3.067, 3.963}^d^

PANT	MAB	0.549 {0.488, 0.620}^d^	0.518 {0.465, 0.597}^d^	0.574 {0.509, 0.650}^d^
	BO	1.262 {1.119, 1.427}^d^	1.170 {1.060, 1.298}^b^	1.247 {1.114, 1.386}^c^
	RES	2.421 {2.177, 2.694}^c^	2.121 {1.933, 2.329}^d^	2.315 {2.102, 2.551}^d^
	ME	11.706 {8.146, 17.416}^d^	6.336 {5.109, 7.937}^d^	5.059 {4.198, 6.075}^d^
	WQ	5.086 {4.392, 5.965}^d^	4.403 {3.813, 5.096}^d^	4.886 {4.188, 5.730}^d^

DAHFP	MAB	0.590 {0.525, 0.663}^d^	0.701 {0.638, 0.776}^d^	0.702 {0.630, 0.782}^d^
	BO	2.123 {1.949, 2.322}^d^	2.375 {2.197, 2.565}^d^	2.277 {2.081, 2.485}^d^
	RES	3.869 {3.572, 4.187}^d^	3.161 {2.947, 3.381}^d^	2.966 {2.730, 3.223}^d^
	ME	11.181 {9.149, 13.657}^d^	10.819 {9.085, 12.903}^d^	8.030 {6.751, 9.725}^d^
	WQ	7.952 {7.176, 8.885}^d^	0.478 {0.339, 0.669}^d^	7.484 {6.475, 8.642}^d^

DBSP	MAB	0.599 {0.537, 0.670}^d^	0687 {0.623, 0.760}^d^	0.690 {0.616, 0.772}^d^
	BO	2.148 {1.964, 2.338}^d^	2.427 {2.250, 2.617}^d^	2.256 {2.065, 2.474}^d^
	RES	3.532 {3.267, 3.819}^d^	3.065 {2.871, 3.283}^d^	3.088 {2.841, 3.374}^d^
	ME	10.884 {8.795, 13.735}^d^	11.655 {9.637, 14.220}^d^	8.241 {6.822, 10.076}^d^
	WQ	7.619 {6.851, 8.501}^d^	6.753 {6.054, 7.572}^d^	7.648 {6.593, 8.978}^d^

PCWTD	MAB	0.605 {0.533, 0.687}^d^	0.782 {0.663, 0.919}^b^	0.713 {0.601, 0.845}^c^
	BO	1.344 {1.195, 1.510}^d^	1.727 {1.522, 1.972}^d^	1.485 {1.308, 1.693}^d^
	RES	2.168 {1.963, 2.393}^d^	2.358 {2.086, 2.658}^d^	2.641 {2.334, 2.977}^d^
	ME	3.527 {2.889, 4.317}^d^	5.529 {4.242, 7.302}^d^	4.135 {3.368, 5.117}^d^
	WQ	2.912 {2.593, 3.270}^d^	3.449 {2.918, 4.113}^d^	5.370 {4.470, 6.476}^d^

SPCWTD	MAB	0.606 {0.531, 0.687}^d^	0.642 {0.543, 0.758}^d^	0.683 {0.575, 0.807}^c^
	BO	1.690 {1.493, 1.918}^d^	2.151 {1.903, 2.427}^d^	1.599 {1.407, 1.812}^d^
	RES	3.597 {3.235, 4.010}^d^	2.640 {2.355, 2.953}^d^	2.796 {2.490, 3.152}^d^
	ME	7.410 {6.006, 9.091}^d^	8.313 {6.520, 10.691}^d^	5.001 {4.095, 6.102}^d^
	WQ	5.614 {5.001, 6.346}^d^	5.293 {4.494, 6.246}^d^	5.788 {4.484, 6.915}^d^

*p*: *p* value; a: *p* > 0.05; b: *p* < 0.05; c: *p* < 0.01; d: *p* < 0.001.

**Table 4:** Comparison of ORs regarding different response variables for years 2006-18 using BLRM.

Response variables	Region/province	PDHS 2006-07	PDHS 2012-13	PDHS 2017-18
		OR (95% CI for OR)	OR (95% CI for OR)	OR (95% CI for OR)
ANC	Punjab (R)	1	1	1
	Sindh	2.327 {2.093, 2.603}^d^	1.024 {0.913, 1.153}^b^	0.498 {0.424, 0.588}^b^
	KPK	0.537 {0.462, 0.621}^d^	0.437 {0.389, 0.493}^d^	0.335 {0.284, 0.398}^c^
	Balochistan	0.785 {0.626, 0.982}^d^	0.125 {0.102, 0.153}^d^	0.104 {0.084, 0.127}^d^

MDDP	Punjab (R)	1	1	1
	Sindh	1.352 {1.214, 1.514}^d^	1.171 {1.067, 1.286}^d^	0.984 {0.883, 1.091}^c^
	KPK	1.068 {0.936, 1.211}^d^	1.236 {1.108, 1.375}^d^	0.790 {0.701, 0.892}^d^
	Balochistan	0.556 {0.444, 0.686}^d^	0.248 {0.193, 0.315}^d^	0.745 {0.621, 0.888}^d^

PANT	Punjab (R)	1	1	1
	Sindh	0.751 {0.660, 0.854}^d^	0.409 {0.372, 0.449}^d^	0.380 {0.342, 0.424}^c^
	KPK	0.561 {0.481, 0.655}^d^	0.444 {0.398, 0.498}^d^	0.335 {0.297, 0.380}^c^
	Balochistan	0.241 {0.183, 0.315}^d^	0.108 {0.087, 0.133}^d^	1.235{1.020, 1.509}^d^

DAHFP	Punjab (R)	1	1	1
	Sindh	1.426 {1.306, 1.549}^d^	1.501 {1.394, 1.618}^d^	1.148 {1.056, 1.256}^c^
	KPK	0.845 {0.758, 0.942}^d^	0.723 {0.660, 0.787}^d^	0.730 {0.662, 0.803}^d^
	Balochistan	0.444 {0.357, 0.541}^d^	0.199 {0.163, 0.238}^d^	0.239 {0.205, 0.278}^d^

DBSP	Punjab (R)	1	1	1
	Sindh	1.319 {1.210, 1.438}^d^	1.388 {1.284, 1.502}^d^	1.194 {1.090, 1.308}^c^
	KPK	1.005 {0.904, 1.116}^a^	0.845 {0.769, 0.926}^d^	0.831 {0.753, 0.9.18}^d^
	Balochistan	0.493 {0.399, 0.604}^d^	0.197 {0.163, 0.234}^d^	0.253 {0.217, 0.295}^d^

PCWTD	Punjab (R)	1	1	1
	Sindh	2.327 {2.093, 2.603}^d^	1.009 {0.888, 1.154}^a^	1.234 {1.069, 1.431}^a^
	KPK	0.537 {0.462, 0.621}^d^	0.311 {0.266, 0.360}^c^	0.382 {0.328, 0.443}^d^
	Balochistan	0.785 {0.626, 0.982}^d^	0.309 {0.240, 0.402}^c^	0.313 {0.241, 0.399}^d^

SPCWTD	Punjab (R)	1	1	1
	Sindh	1.761 {1.574, 2.971}^d^	1.272 {1.117, 1.441}^a^	1.082 {0.947, 1.244}^c^
	KPK	0.714 {0.608, 0.838}^d^	0.536 {0.459, 0.625}^c^	0.379 {0.325, 0.444}^d^
	Balochistan	0.514 {0.383, 0.689}^d^	0.138 {0.095, 0.198}^d^	0.246 {0.186, 0.325}^d^

*p*: *p* value; a: *p* > 0.05; b: *p* < 0.05; c: *p* < 0.01; d: *p* < 0.001.

**Table 5:** Comparison of ORs regarding different response variables for years 2006-18 using classical logistic regression model.

Response variables	Explanatory variables	PDHS 2006-07	PDHS 2012-13	PDHS 2017-18
		OR (95% CI for OR)	OR (95% CI for OR)	OR (95% CI for OR)
ANC	MAB	0.558 {0.483, 0.643}^d^	0.498 {0.434, 0.571}^d^	0.494 {0.414, 0.592}^d^
	BO	1.963 {1.685, 2.293}^d^	2.240 {1.927, 2.614}^d^	2.734 {2.184, 3.465}^d^
	RES	3.103 {2.726, 3.538}^d^	3.586 {3.126, 4.127}^d^	3.607 {2.982, 4.398}^d^
	ME	17.763 {10.621, 32.651}^d^	14.504 {9.443, 23.773}^d^	34.212 {15.810, 95.785}^d^
	WQ	9.679 {7.726, 12.287}^d^	13.314 {9.907, 18.398}^d^	11.053 {7.396, 17.466}^d^

MDDP	MAB	0.607 {0.523, 0.703}^d^	0.741 {0.649, 0.847}^d^	0.983 {0.849, 1.139}^a^
	BO	1.444 {1.257, 1.659}^d^	1.539 {1.371, 1.728}^d^	1.517 {1.338, 1.723}^d^
	RES	2.459 {2.191, 2.762}^d^	2.111 {1.909, 2.336}^d^	1.661 {1.494, 1.849}^d^
	ME	6.990 {5.284, 9.405}^d^	5.129 {4.238, 6.247}^d^	3.948 {3.296, 4.759}^d^
	WQ	4.602 {3.965, 5.354}^d^	3.320 {2.915, 3.789}^d^	3.491 {3.004, 4.072}^d^

PANT	MAB	0.549 {0.476, 0.633}^d^	0.518 {0.454, 0.591}^d^	0.574 {0.495, 0.665}^d^
	BO	1.262 {1.093, 1.458}^d^	1.172 {1.038, 1.324}^b^	1.244 {1.091, 1.422}^c^
	RES	2.426 {2.143, 2.749}^c^	2.122 {1.901, 2.372}^d^	2.315 {2.055, 2.612}^d^
	ME	11.816 {7.704, 19.232}^d^	6.346 {4.908, 8.355}^d^	5.054 {4.046, 6.394}^d^
	WQ	5.102 {4.257, 6.150}^d^	4.399 {3.727, 5.223}^d^	4.893 {4.058, 5.948}^d^

DAHFP	MAB	0.591 {0.513, 0.679}^d^	0.702 {0.623, 0.789}^d^	0.699 {0.614, 0.797}^d^
	BO	2.124 {1.916, 2.354}^d^	2.380 {2.180, 2.599}^d^	2.274 {2.049, 2.527}^d^
	RES	3.867 {3.518, 4.252}^d^	3.156 {2.904, 3.431}^d^	2.967 {2.690, 3.276}^d^
	ME	11.301 {8.969, 14.409}^d^	10.867 {8.853, 13.488}^d^	8.075 {6.545, 10.086}^d^
	WQ	7.962 {7.041, 9.020}^d^	0.476 {0.311, 0.712}^d^	7.472 {6.298, 8.931}^d^

DBSP	MAB	0.601 {0.525, 0.686}^d^	0687 {0.611, 0.772}^d^	0.688 {0.603, 0.787}^d^
	BO	2.150 {1.941, 2.381}^d^	2.425 {2.217, 2.653}^d^	2.257 {2.025, 2.519}^d^
	RES	3.535 {3.219, 3.883}^d^	3.070 {2.822, 3.343}^d^	3.094 {2.792, 3.435}^d^
	ME	10.957 {8.580, 14.192}^d^	11.638 {9.304, 14.763}^d^	8.274 {6.602, 10.524}^d^
	WQ	7.622 {6.714, 8.673}^d^	6.763 {5.931, 7.739}^d^	7.638 {6.360, 9.257}^d^

PCWTD	MAB	0.605 {0.519, 0.704}^d^	0.780 {0.644, 0.945}^b^	0.711 {0.581, 0.872}^c^
	BO	1.344 {1.168, 1.545}^d^	1.725 {1.484, 2.008}^d^	1.487 {1.274, 1.739}^d^
	RES	2.168 {1.931, 2.433}^d^	2.356 {2.039, 2.726}^d^	2.639 {2.277, 3.066}^d^
	ME	3.531 {2.802, 4.478}^d^	5.525 {4.054, 7.715}^d^	4.169 {3.288, 5.349}^d^
	WQ	2.909 {2.533, 3.344}^d^	3.469 {2.830, 4.284}^d^	5.392 {4.333, 6.777}^d^

SPCWTD	MAB	0.541 {0.450, 0.647}^d^	0.642 {0.527, 0.779}^d^	0.681 {0.556, 0.833}^c^
	BO	1.691 {1.458, 1.958}^d^	2.155 {1.865, 2.492}^d^	1.487 {1.274, 1.739}^d^
	RES	3.598 {3.179, 4.075}^d^	2.630 {2.295, 3.016}^d^	2.639 {2.277, 3.066}^d^
	ME	7.442 {5.871, 9.497}^d^	8.417 {6.254, 11.572}^d^	4.169 {3.288, 5.349}^d^
	WQ	5.631 {4.881, 6.502}^d^	5.298 {4.356, 6.484}^d^	5.392 {4.333, 6.677}^d^

*p*: *p* value; a: *p* > 0.05; b: *p* < 0.05; c: *p* < 0.01; d: *p* < 0.001.

**Table 6:** Comparison of odds ratios regarding ANC for years 2006-18 using Bayesian logistic regression.

Factors	2006-07	2012-13	2017-18
*Mother age at birth*			
<20	1.504 {1.240, 1.806}^d^	2.085 {1.727, 2.558}^d^	1.617 {1.269, 2.058}^c^
20-34	1.835 {1.629, 2.077}^d^	1.997 {1.787, 2.241}^d^	2.060 {1.778, 2.382}^d^
35-49 (R)	1	1	1
*Birth order*			
1	2.791 {2.403, 3.253}^d^	4.995 {3.453, 4.599}^d^	5.683 {4.614, 7.116}^d^
2-3	2.011 {1.782, 2.266}^d^	2.710 {2.419, 3.040}^d^	3.262 {2.770, 3.813}^d^
4-5	1.297 {1.151, 1.471}^d^	1.760 {1.565, 1.983}^d^	2.060 {1.762, 2.405}^d^
6+ (R)	1	1	1
*Residence*			
Urban (R)	1	1	1
Rural	0.322 {0.289, 0.358}^d^	0.278 {0.246, 0.314}^d^	0.277 {0.234, 0.325}^d^
*Mother education*			
No education	0.040 {0.024, 0.066}^d^	0.043 {0.029, 0.061}^d^	0.017 {0.008, 0.034}^d^
Primary	0.094 {0.057, 0.147}^d^	0.125 {0.081, 0.184}^d^	0.073 {0.032, 0.145}^d^
Middle	0.181 {0.092, 0.321}^d^	0.291 {0.184, 0.448}^d^	0.145 {0.066, 0.292}^d^
Secondary	0.292 {0.105, 0.288}^d^	0.587 {0.361, 0.926}^a^	0.145 {0.062, 0.297}^d^
Higher (R)	1	1	1
*Wealth quintile*			
Lowest	0.051 {0.041, 0.063}^d^	0.036 {0.027, 0.046}^d^	0.037 {0.025, 0.052}^d^
Second	0.082 {0.066, 0.102}^d^	0.056 {0.042, 0.072}^d^	0.075 {0.051, 0.105}^d^
Middle	0.140 {0.113, 0.173}^d^	0.115 {0.086, 0.151}^d^	0.206 {0.139, 0.295}^d^
Fourth	0.247 {0.197, 0.308}^d^	0.233 {0.171, 0.312}^d^	0.401 {0.262, 0.593}^d^
Highest (R)	1	1	1
*Province*			
Punjab (R)	1	1	1
Sindh	2.327 {2.093, 2.603}^d^	1.024 {0.913, 1.153}^b^	0.498 {0.424, 0.588}^b^
KPK	0.537 {0.462, 0.621}^d^	0.437 {0.389, 0.493}^d^	0.335 {0.284, 0.398}^c^
Balochistan	0.785 {0.626, 0.982}^d^	0.125 {0.102, 0.153}^d^	0.104 {0.084, 0.127}^d^

a: *p* > 0.05; b: *p* < 0.05; c: *p* < 0.01; d: *p* < 0.001.

## Data Availability

The data is available in the published reports of Pakistan Demographic and Health Surveys (PDHS) conducted in 2006-07, 2012-13, and 2017-18. These reports are available at: http://nhsrc.pk/dashboards/pdhsselect.html.
